The article "Relaxin-3 Ameliorates Diabetic Cardiomyopathy by Inhibiting Endoplasmic Reticulum Stress" was retracted in 2023. Reasons: signs of a paper mill; compromised peer review; unreliable results or conclusions.

# Relaxin-3 Ameliorates Diabetic Cardiomyopathy by Inhibiting Endoplasmic Reticulum Stress

**DOI:** 10.1155/2022/9380283

**Published:** 2022-09-27

**Authors:** Li-ya Pan, Xiao-hui Zhang, Wu-jie Xia, Jia-lin Pan

**Affiliations:** ^1^Department of Cardiology, The Second Affiliated Hospital and Yuying Children's Hospital of Wenzhou Medical University, Wenzhou 325000, China; ^2^Department of Cardiology, The First Affiliated Hospital of Harbin Medical University, Harbin 150001, China

## Abstract

**Background:**

This study is aimed at investigating whether relaxin-3 exhibits protective effects against cardiomyopathy in diabetic rats by suppressing ERS.

**Methods:**

Eighty male SD rats were randomly divided into two groups: controls (*n* = 20) and diabetes (*n* = 60). The streptozotocin-treated rats were randomly divided into three groups: diabetic group (DM), low-dose relaxin-3 group (0.2 *μ*g/kg/d), and high-dose relaxin-3 group (2 *μ*g/kg/d). The myocardial tissues and collagen fiber were observed by hematoxylin and eosin (H&E) and Masson staining. Serum brain natriuretic peptide (BNP), troponin (TNI), myoglobin, interleukin (IL-17), interleukin (IL)-1*α*, and tumor necrosis factor (TNF)-*α* were determined by ELISA. The protein expression of glucose regulatory protein 78 (GRP78) and C/EBP homologous protein (CHOP) in the heart tissue of each group was detected by Western blot analysis.

**Results:**

(1) HE and Masson staining indicated that relaxin-3 could attenuate myocardial lesions and myocardial collagen volume fraction. (2) BNP, TnI, and myoglobin in the DM group at four and eight weeks were significantly higher than in the controls (*P* < 0.01). The relaxin-3-treated groups showed significantly reduced serum BNP, TnI, and myoglobin levels compared with the DM group (*P* < 0.05). (3) IL-17, IL-1*α*, and TNF-*α* levels in the DM rats at 4 weeks were higher than in the controls (*P* < 0.05). Low or high dose of relaxin-3-treated groups showed reduced serum IL-17 and TNF-*α* levels compared with the DM group at four and eight weeks (*P* < 0.05). (4) CHOP and GRP78 protein expression was increased in the DM group at four and eight weeks compared with the controls (*P* < 0.01), and small and large doses of relaxin-3 significantly reduced GRP78 and CHOP protein expression.

**Conclusions:**

Exogenous relaxin-3 ameliorates diabetic cardiomyopathy by inhibiting ERS in diabetic rats.

## 1. Introduction

Diabetic cardiomyopathy is a type of myocardial disease in diabetes mellitus patients, independent of hypertension and coronary artery disease. It is characterized by diastolic and systolic dysfunction, which can lead to congestive heart failure. Numerous mechanisms have been proposed to contribute to the development of diabetic cardiomyopathy including metabolic disturbances, myocardial fibrosis, myocardial cell apoptosis, small vessel disease, oxidative stress, and inflammation. Recently, endoplasmic reticulum stress (ERS) has been reported to play a critical role in diabetic cardiomyopathy [1]. In diabetes complications, various factors such as ischemia, hypoxia, oxidative stress, or disturbance of calcium homeostasis can interfere with ER function, leading to accumulation of unfolded or incorrectly folded proteins, and subsequent activation of the corresponding signal transduction pathways such as ER Ca^2+^ buffering, to restore the endoplasmic reticulum homeostasis [2]. If prolonged, the ER stress responses, as well as protein and lipid turnover, disrupt many cardiac functions, including energy metabolism and cardiogenesis, cause cardiac insulin resistance, and ultimately result in cardiomyopathy and heart failure [3]. Therefore, ERS is a potential therapeutic target for diabetic cardiomyopathy; regulation of ERS may reduce the risk of myocardial injury and prevent complications induced by diabetes [3].

Relaxin-3 is one member of the relaxin peptide family that was first discovered in the brain in 2002. Relaxin-3 has been demonstrated to have cardiovascular protective effects [4]. Furthermore, our research group has revealed that relaxin-3 inhibited high glucose-induced apoptosis in high-glucose-treated neonatal rat ventricular myocytes, mediated by suppressing the extrinsic and intrinsic pathways of apoptosis and ERS [5]. Based on these findings and considering that ERS is an important factor in the pathogenesis of cardiomyopathy, we hypothesized that relaxin-3 can ameliorate myocardial injury in diabetes complications. Therefore, in this study, we investigated the effects of relaxin-3 on diabetic cardiomyopathy in streptozotocin- (STZ-) induced diabetic rats and whether the cardioprotective effects of relaxin-3 were mediated through inhibition of ERS.

## 2. Materials and Methods

### 2.1. Materials

Relaxin-3 was from Phoenix Pharmaceuticals (Belmont, CA, USA), Streptozotocin was obtained from Sigma Chemical Co. (St. Louis, MO, USA). Goat polyclonal antiglucose regulatory protein 78 (GR P78) and anti-C/EBP homologous protein (CHOP) were obtained from Abcam (Cambridge, UK), and ELISA kits were obtained from Jiancheng Co. (Nanjing, China).

### 2.2. Animals and Reagents

The study protocol was approved by the Animal Care and Use Committee of the first affiliated hospital of Harbin Medical University. Eighty male Sprague Dawley (SD) rats (250-300 g) were purchased from the Animal Center of the Second Affiliated Hospital of Harbin Medical University. All the rats were acclimatized to the environment and given water and a normal rat diet for a week before the start of the experiment. Eighty male SD rats were randomly divided into two groups: controls (*n* = 20) and diabetes (*n* = 60). Diabetic models were established by a single intraperitoneal injection of STZ at a dose of 65 mg/kg. Three and seven days after STZ injection, the rats' venous blood glucose levels were measured and the rats with blood glucose higher than 16.6 mmol/L were considered successful diabetic models. The STZ-treated rats were divided into three groups randomly: diabetic (DM) group, low-dose relaxin-3 group (0.2 *μ*g/kg/d), and high-dose relaxin-3 group (2 *μ*g/kg/d). The rats were treated with subcutaneous relaxin-3 injection for two weeks and two and six weeks after the diabetic models were established. Then, heart tissue samples were collected at four and eight weeks.

### 2.3. Hematoxylin and Eosin and Masson Staining

The apical tissues were immersed in 4% paraformaldehyde, embedded in paraffin, and serially cut. Then, they were stained with hematoxylin and eosin (H&E) and Masson to observe the myocardial tissues and collagen fiber.

### 2.4. Determination of Troponin and Brain Natriuretic Peptide by ELISA

Blood samples obtained from the abdominal aorta were centrifuged at 3500r for 10 min. The supernatant was collected for determination of cardiac troponin (cTn)-I and brain natriuretic peptide (BNP) levels by ELISA.

### 2.5. Determination of Myoglobin

According to the Elz and Nayler method [6], 100 *μ*L of the rats' serum samples was centrifuged at 3000r for 5 min and placed in a microplate reader at a wavelength of 410 nm (the reading of distilled water was zero). Myoglobin content was determined as (mg/mL) = 0.187 × OD value.

### 2.6. Determination of IL-17, IL-1*α*, and TNF-*α*

50 *μ*L of the rats' serum samples was collected, and the content of IL-17, IL-1*α*, and TNF-*α* was measured by ELISA.

### 2.7. Western Blot Analysis

After the rats were killed, the myocardial tissue was collected and processed according to the manufacturer's instructions. The primary antibodies and dilutions were antiglucose regulatory protein 78 (GRP78), 1 : 1000, anti-C/EBP homologous protein (CHOP), 1 : 500, and anti-*β*-actin (1 : 1000). Secondary anti-rabbit or anti-mice antibodies were used at a dilution of 1 : 2000. The results were visualized using enhanced chemiluminescence detection kits and were analyzed using the Quantity One software.

### 2.8. Statistical Analysis

GraphPad Prism (version 5.0) was used to analyze data. The results were expressed as mean ± SD. For more than two groups, we used the ANOVA, followed by a Newman-Keuls multiple comparison test, and *P* < 0.05 was considered statistically significant.

## 3. Results

### 3.1. Effects of Relaxin-3 on Myocardial Pathological Abnormalities in Diabetic Rats

On haematoxylin and eosin staining, myocardial cells in the control group at four and eight weeks appeared to be more compact and arranged in an orderly manner. However, in the DM group, disorderly arranged myocardial cells and irregular nuclei and cardiomyocyte atrophy were observed. Furthermore, rupture of myocardial fibers was observed at eight weeks in the DM group. Relaxin-3 attenuated the above myocardial injury, especially in rats that were administered high doses of relaxin-3.

After the Masson staining, in the control group at four and eight weeks, orderly cardiomyocytes and only a little collagen deposition were observed. In the DM group, at four weeks, myocardial cells showed an irregular arrangement and increased interstitial collagen fibers, and a large amount of collagen deposition was observed at eight weeks. Relaxin-3 treatment reduced the collagen fibers in the intercellular and perivascular space, especially in the high-dose relaxin-3 group (Figures 1 and 2).

### 3.2. Relaxin-3 Ameliorates Myocardial Injury in Diabetic Rats

BNP, TnI, and myoglobin in the DM group at four weeks were significantly higher than in the controls (*P* < 0.01). BNP and TnI were significantly increased in the DM group at 8 weeks (*P* < 0.01). A similar trend was observed with myoglobin (*P* < 0.05). Treatment with relaxin-3 significantly reduced serum BNP, TnI, and myoglobin levels in both of the treatment groups compared with the DM group at four and eight weeks (*P* < 0.05) (Figure 3).

### 3.3. Relaxin-3 Inhibited Inflammation in the Myocardial Tissues in Diabetic Rats

IL-17, IL-1*α*, and TNF-*α* in DM rats at four weeks were higher in the DM rats than in the controls (*P* < 0.05), and there was upregulated expression of IL-17 in the DM rats at eight weeks (*P* < 0.05), but the difference in the expression of IL-1*α* and TNF-*α* between the groups had no statistical significance (*P* > 0.05). Relaxin-3 at either small or large dose reduced serum IL-17 and TNF-*α* levels compared with the DM group at four and eight weeks (*P* < 0.05). And both doses of relaxin-3 reduced IL-1*α* in the DM rats at four weeks (*P* < 0.01), but there was no significant difference observed in the DM rats at eight (*P* > 0.05) (Figure 4).

### 3.4. Relaxin-3 Inhibited ERS in the Myocardial Tissues of Diabetic Rats

CHOP and GRP78 were significantly increased in the DM group at four and eight weeks compared with the controls (*P* < 0.01); after the treatment of relaxin-3, significantly decreased GRP78 and CHOP protein expression was observed compared with the DM group, particularly in the high dose of relaxin-3 group (Figure 5).

## 4. Discussion

Diabetic cardiomyopathy (DCM), independent of coronary heart disease and hypertension, was first discovered by Rubler et al. [7]. Recent studies have shown that ERS plays an important role in the development of diabetic cardiomyopathy. Therefore, it is a potential therapeutic target for cardiomyopathy.

Relaxin-3 is one of the most important endogenous peptides that can inhibit fibrosis and have cardiovascular protective effects. Zhang et al. found that relaxin-3 was protective against myocardial ischemia injury induced by isoproterenol [8]. In our study, we established diabetic models with 65 mg/kg STZ injection. The rats' blood glucose was significantly increased and maintained at a high level (blood glucose over 16.6 mmol/L). After STZ injection for one week, the diabetic rats showed polydipsia, polyuria, or polyphagia symptoms. Moreover, their fur was noticeably cluttered, and they lost weight.

Studies have shown that an increase in inflammation in diabetic myocardial tissue may be involved in the pathophysiology of diabetic cardiomyopathy [9]. Inflammatory factors and diabetic cardiomyopathy are closely related. Metabolic disorders such as glycometabolism and lipid metabolism may cause chronic inflammation. Consequently, inflammatory factors accumulate in the myocardial cells, triggering myocardial cell apoptosis [10]. TNF-*α*, IL-17, and IL-1*α* are overexpressed in diabetes patients. Excess TNF-*α* can mediate immune response, induce cell apoptosis, inhibit myocardial contraction, and participate in myocardial remodeling [11]. Bryant found that TNF-*α* overexpression in transgenic mice caused heart enlargement, heart dysfunction, and myocardial fibrosis [12]. IL-17 activated NF-*κ*B and stimulated the proinflammatory factors such as IL-6, TNF-*α*, and GM-CSF to induce inflammation and then participate in the development of diabetic cardiomyopathy [13]. IL-1 which promoted myocardial hypertrophy, induced myocardial cell apoptosis and inhibited myocardial contractions which are key factors in the pathogenesis of heart failure [14]. In our study, inflammatory factors increased in the diabetic rats' serum at four weeks compared with the controls. After the treatment with relaxin-3, the number of inflammatory factors reduced, which indicated that relaxin-3 inhibited the expression of inflammatory factors. Chronic inflammation can lead to fibrosis and tissue remodeling. However, there was no significant difference in the inflammatory factors between the control group and diabetic rats at eight weeks. On the other hand, disordered myocardial tissues and a large amount of collagen deposition were seen in DM rats at 8 weeks. Meanwhile, the relaxin-3 treatment group showed significantly reduced serum BNP, TnI, and myoglobin levels compared with the DM group. Relaxin-3 might attenuate diabetic myocardial injury by inhibiting some inflammatory factors.

ERS is involved in various cardiovascular diseases, such as heart failure, diabetic cardiomyopathy, and hypertension [15, 16]. ER stress is aimed initially at compensating for damage; when in excess or prolonged, it can eventually trigger cell death of ER stress. The main signal transduction pathways of ERS include protein kinase R-like ER kinase (PERK), activating transcription factor 6 (ATF6), and inositol-requiring enzyme type 1 (IRE1) pathways [17]. GRP78 is a classic marker of ERS; the upregulation of GRP78 expression means the activation of ERS. Normally, the expression of CHOP is low, but when stimulated, the ERS-associated pathways such as PERK, ATF-6, and IRE1 pathways can all activate CHOP and eventually led to apoptosis. ERS is one of the important mechanisms of diabetic cardiomyopathy [18, 19]. In 1985, Jackson et al. demonstrated ultrastructural evidence of swelling and dilation of ER in the diabetic myocardium model. These findings suggest that ER stress is a potential therapeutic target for diabetic cardiomyopathy [20]. In 2007, Li et al. found that GRP78 and caspase-12 were upregulated in an STZ-induced type I diabetic rat model. The ER stress-associated apoptosis may be a factor in the pathogenesis of diabetic cardiomyopathy [21]. Previous studies have shown that relaxin-3 can inhibit high-glucose-induced apoptosis in high-glucose-treated neonatal rat ventricular myocytes by the activation of the extrinsic and intrinsic pathways of apoptosis and ERS. In this study, compared with the control group, the expression of GRP78 and CHOP in the myocardial tissues of the diabetic rats increased, suggesting that endoplasmic reticulum stress was involved in the myocardial injury in diabetic rats. After exogenous relaxin-3 treatment, both low and high doses, the expression of GRP78 and CHOP decreased in the treatment group compared with the DM group. These findings suggest that relaxin-3 may downregulate the expression of GRP78 and CHOP by inhibiting ERS to ameliorate myocardial injury in diabetic rats.

This study has limitations. While other tests such as echocardiography and analysis are important in strengthening our findings; in this study, they were not conducted. Therefore, in the future, more tests and further analysis should be included to prove these findings.

## 5. Conclusion

In summary, our findings indicate that exogenous relaxin-3 ameliorates myocardial injury in diabetic rats which may due to its inhibition of ER stress and inflammation. Therefore, our results suggest a novel therapeutic strategy for ameliorating myocardial injury induced by diabetes.

## Figures and Tables

**Figure 1:** HE and Masson staining of myocardium in rats at 4 weeks. (a) Hematoxylin and eosin staining (200x magnification, scale bar 100 *μ*m); (b) Masson staining (200x magnification, scale bar 100 *μ*m).

**Figure 2:** HE and Masson staining of myocardium in rats at 8 weeks. (a) Hematoxylin and eosin staining (200x magnification, scale bar 100 *μ*m); (b) Masson staining (200x magnification, scale bar 100 *μ*m).

**Figure 3:** Relaxin-3 inhibited the expression of BNP, TNI, and myoglobin in the serum of DM rats. (a) Relaxin-3 inhibited the expression of BNP in the serum of DM rats. (b) Relaxin-3 inhibited the expression of TNI in the serum of DM rats. (c) Relaxin-3 inhibited the expression of myoglobin in the serum of DM rats. ^∗^*P* < 0.05 vs. control, ^∗∗^*P* < 0.01 vs. control, ^#^*P* < 0.05 vs. DM, ^##^*P* < 0.01 vs. DM.

**Figure 4:** Relaxin-3 inhibited the expression of IL-17, IL-1*α*, and TNF-*α* in the serum of DM rats. (a) Relaxin-3 inhibited the expression of IL-17 in the serum of the DM rats. (b) Relaxin-3 inhibited the expression of IL-1*α* in the serum of the DM rats. (c) Relaxin-3 inhibited the expression of TNF-*α* in the serum of the DM rats. ^∗^*P* < 0.05 vs. control, ^∗∗^*P* < 0.01 vs. control, ^#^*P* < 0.05 vs. DM, ^##^*P* < 0.01 vs. DM.

**Figure 5:** Relaxin-3 inhibited ERS in the myocardial tissues of DM rats. (a) GRP78 and CHOP protein expression was analyzed by Western blot. (b) Analysis of the GRP78 protein level (GRP78/*β*-actin). (c) Analysis of the CHOP protein level (CHOP/*β*-actin). ^∗^*P* < 0.05 vs. control, ^∗∗^*P* < 0.01 vs. control, ^#^*P* < 0.05 vs. DM, ^##^*P* < 0.01 vs. DM.

## Data Availability

The data used to support the findings of this study are available from the corresponding author upon request.
